# Research on the Mining of Intangible Cultural Heritage Digital Resources in the Manual Online Teaching System of Preschool Education

This article has been retracted.

**DOI:** 10.1155/2022/2136597

**Published:** 2022-04-23

**Authors:** Zhao Jun, Xingping Li

**Affiliations:** Ganzhou Teachers College, Jiangxi 341000, China

## Abstract

Our country's international status as a cultural power has been further enhanced, and the protection of intangible cultural heritage containing the essence of traditional culture is also gradually being carried out. In addition, with the rapid development of the digital environment, the public's cultural needs continue to grow, and the contradiction between the supply and demand of public digital cultural services continues to intensify. Converting intangible cultural heritage into digital form for protection and providing resource services for the public has become an important trend in the protection and inheritance of intangible cultural heritage at home and abroad, and it is also an inevitable requirement to solve the contradiction between supply and demand. Improving public cultural services is one of the key projects. At present, our country's research and practice of intangible cultural heritage digitization and services are also in progress, but there is no research on intangible cultural heritage digital resource services and system construction from the perspective of information service elements. Based on the digital resource service of intangible cultural heritage, the manual course is one of the main skill courses for preschool education majors. At this stage, the short class hours of manual courses, the lack of class hours, the low utilization rate of teaching materials, and the disconnection between the content and the needs of the kindergarten are all problems that need to be solved at present. Just relying on cross-references between schools, the manual knowledge and skills mastered by graduates are not comprehensive enough to complete the manual tasks assigned by the kindergarten. This paper implements the concept of intangible cultural heritage and hopes that by studying the manual knowledge and skills that today's kindergarten teachers need to possess, the content of existing manual courses can be adjusted in a targeted manner, so that the electronic culture dissemination of manual curriculum resources for preschool education is more reasonable, meeting the requirements of kindergarten teachers in terms of manual knowledge and skills.

## 1. Introduction

The Chinese nation has a long history, and its excellent traditional culture is extensive and profound. The land of Guangxiang in China has nurtured a rich variety of precious and wonderful intangible cultural heritage (hereinafter referred to as “intangible cultural heritage”). These intangible cultural heritages are the spiritual essence of Chinese culture. Protecting and making good use of them is of great significance to enhancing national unity, developing cultural self-confidence, meeting people's growing needs for a better life, and maintaining world cultural diversity and creativity [1, 2]. However, due to our country's vast territory and abundant resources and the variety and quantity of intangible cultural heritage, the current protection work still cannot meet the needs of intangible cultural heritage protection, and some intangible cultural heritage items have not been included in the scope of protection. The disappearance of intangible cultural heritage such as the destruction of the original environment of intangible cultural heritage and the lack of successors of intangible cultural heritage is not an exception. The protection and inheritance of national cultural treasures on the verge of extinction have become an urgent task for the country and the nation [3–5].

The construction of intangible cultural heritage digital resource services is also an inevitable choice to improve public cultural services. The people's material living standard is prosperous, and the demand for cultural and artistic accomplishment is even stronger. It is necessary to provide rich spiritual and cultural services to meet the new demand for culture. In his report on the future construction of socialist culture with Chinese characteristics, General Secretary Xi Jinping emphasized the need to strengthen cultural self-confidence, improve the construction of the government's public cultural service system, and attach importance to the development and dissemination of the traditional cultural heritage of the Chinese nation [6–8]. In recent years, our country's public cultural services have developed rapidly, but there are still problems such as insufficient investment, unbalanced development, and low quality. In view of the diversification of the main body of the people's cultural resource demand, the integration of content, the diversification of carrier forms, and the efficient utilization of the people's cultural resources, it is necessary for the country and the government to provide rich, convenient, and professional public digital cultural services in line with the development of the times and to meet the needs of users. Libraries, museums, archives, and other institutions, as the main public cultural service institutions, provide intangible cultural heritage digital resource services to expand the scope of public cultural services and promote the improvement of public cultural services in the context of the big data era [9, 10]. It can be seen that under the background of the severe situation of intangible cultural heritage protection and the growing spiritual and cultural needs, the construction of intangible cultural heritage digital resource service system has become an important task of the current government and public cultural institutions [10–12].

Like foreign countries, domestic scholars have also explored the application and practical research of digital technology in the protection of intangible cultural heritage from the technical dimension. Riji combined AR technology and intangible cultural heritage protection to explore the theoretical and practical value of augmented reality technology in the development of intangible cultural heritage protection. Tan Guoxin and Sun Chuanming aimed at the problems faced by the digital protection and dissemination of intangible cultural heritage, and guided by the theory of information space, they realized the specific application research of the digital development protection of the intangible cultural heritage project “Saye Erho” based on 3D technology. Wang Meng and Xu Xin combined the theme map model to visualize the historical origins, inheritance context, genre development, and other characteristics of Peking Opera, Kunqu Opera, and other drama intangible cultural heritage. In terms of the organization of intangible cultural heritage digital resources, Tan Guoxin, Zhai Shanshan, Xu Xin, and others analyzed and summarized the existing intangible cultural heritage metadata standards and semantic organization description, respectively, and put forward research insights on the organization of intangible cultural heritage digital resources [13, 14].

The construction and service of intangible cultural heritage digital resources in China are sporadic in theory and practice and are still in the initial stage of development. Facing the increasingly severe demise of intangible cultural heritage, whether it is from the perspective of cultural heritage protection, inheritance, and development or the improvement of public digital cultural services, the study of intangible cultural heritage digital resource services itself contains theoretical and practical research significance. Using advanced digital technology to protect and disseminate intangible cultural heritage resources and build an advanced and complete intangible cultural heritage digital resource service system not only breeds a good development environment for the theory and practice of intangible cultural heritage protection in our country but also promotes the innovation and development of public cultural services. Ultimately achieve the development goal of cultural self-confidence and promote the great prosperity and development of socialist cultural construction [15–17].

The establishment of the preschool education major in higher vocational colleges provides professional and skilled talents for early childhood education. As a professional skill course, hand-made courses are actually used in most places in kindergarten teaching. Its practical application value is the most direct. Compared with other skill courses, hand-made courses are more maneuverable and practical. However, compared with other skill courses, there are still many problems and challenges in curriculum construction and development. For example, the construction and development of hand-made courses in preschool education in some higher vocational schools is slow, and the quality of courses is not good. Students' operational skills and practical skills are poorly cultivated and applied. These problems make it difficult for students to use flexibly in practical skills operation and can not well adapt to the needs of work development. The research on hand-made courses mostly stays in the summary of teaching problems and experience, and there is less research on the hand-made courses themselves [18–20].

This paper compares and studies the current situation and cases of intangible cultural heritage digital resource services at home and abroad and concludes that the service principle is to focus on user needs, establish a resource co-construction and sharing mechanism under the leadership of the government and cross-institutional and cross-regional collaboration, enrich the quantity and quality of resources, and focus on new experience and inspiration, application of new methods, and establishment of a complete technical standard system for intangible cultural heritage digital resource services. Under the guidance of information service theory, new public from three aspects: technology service theory, and system theory, this paper defines and analyzes the components of our country's intangible cultural heritage digital resource service system from the perspective of information service elements: service goals, service subjects, service resources, and standards. Four elements are proposed, and the construction ideas and model framework of our country's intangible cultural heritage digital resource service system based on element analysis are proposed. The paper discusses the management mechanism of the service system and the three security systems of policies and funds. From meeting the needs of the public as the service goal, speed up the construction and integration of service resources, optimize the management mechanism led by the government and encourage multi-party participation, build a digital technology system for intangible cultural heritage with unified scientific standards, and improve the multifaceted security system [21–24].

On the basis of understanding the concept and theoretical background, this paper compares and studies the service cases of intangible cultural heritage digital resources at home and abroad, sorts out the constituent elements and relationships of our country's intangible cultural heritage digital resource service system, and builds a model of China's intangible cultural heritage digital resource service system based on element analysis. Build ideas and implementation paths. Then, under this system, through the investigation of the current status of intangible cultural heritage digital resource services and user needs, an optimized implementation strategy is proposed for the current intangible cultural heritage digital resource service system.

This paper is organized as follows.  Section 1 introduces the research background of this paper in detail and expounds the research status of domestic and foreign intangible cultural heritage digital resource services.  Section 2 expounds and defines the two concepts of intangible cultural heritage digital resources and public digital cultural services involved in this paper and makes a basic introduction to the main research theories applied in this paper.  Section 3 selects representative cases of intangible cultural heritage digital resource service at home and abroad for analysis and research, summarizes the characteristics of intangible cultural heritage digital resource service at home and abroad, and provides inspiration for the next step in the study of the intangible cultural heritage digital resource service system.  Section 4 deals with the construction of our country's intangible cultural heritage digital resource service system based on element analysis.  Section 5 summarizes the research results and current deficiencies of this paper and puts forward prospects for future research.

The paper has the following innovative contributions:

1. This paper carries out research on the service and system construction of intangible cultural heritage digital resources from the perspective of information service elements.
2. Based on the digital resource service of intangible cultural heritage, the study and practice of handicraft courses are carried out.
3. This paper implements the concept of intangible cultural heritage and hopes to adjust the content of the existing manual courses in a targeted manner by studying the manual knowledge and skills that teachers need in today's kindergartens, so as to make the manual curriculum resources of electronic culture dissemination of preschool education more reasonable.

## 2. Research on Intangible Cultural Heritage

As a core skill course in the art skills course, the handcraft course plays an important role in the art and children's art creation, and the play teaching aids and kindergarten environment creation courses. It belongs to the basic course of handicraft courses. Through the analysis and understanding of the current situation of the five-year consistent preschool education hand-made curriculum in higher vocational colleges, it provides a theoretical basis for the hand-made curriculum for preschool education majors and provides a theoretical basis for the development of hand-made courses, as follows.

(1) $$\begin{array}{c} t=\frac{\sum_{i=1}^{n}t_{i}/dd_{i}^{2}}{\sum_{i=1}^{n}1/dd_{i}^{2}}. \end{array}$$

First of all, through the research of manual curriculum setting, improve the scientific nature of curriculum setting, thereby promoting the progress of teaching efficiency. Finally, through the research on regional preschool education manual courses, in order to strengthen the characteristics of preschool education in this region and promote the development of preschool education in higher vocational colleges, the formula is as follows:

(2) $$\begin{array}{c} d_{ii}={\left(X-X_{ii}\right)}^{1/k}+{\left(Y-Y_{ii}\right)}^{1/k}. \end{array}$$

For the definition of the concept of preschool education, the main focus is on the age division of educational objects. Liang Zhisang proposed in “Preschool Education”: The age object of today's preschool education research should be children from birth to preschool. It can be subdivided into two educational age stages, namely, 0–3 years old and 3–6 years old early childhood education. The age of preschool education objects has shown a gradual downward trend, which is an inevitable choice for social development. Zheng Zheng Jiancheng pointed out in “Preschool Education”: preschool education refers to the education implemented for children aged 0–6. To sum up, according to the needs of the research, this study is mainly aimed at the education of 3–6-year-old children in kindergarten. Therefore, the concept of preschool education is defined as the education of children (3–6 years old) in kindergarten. The purposeful and systematic education is implemented to promote their physical and mental development, as follows:

(3) $$\begin{array}{c} dd_{i}=-\int X_{i}\text{ln}\frac{X_{i}i}{Y_{i}i}\text{dx}. \end{array}$$

Preschool teachers are an important part of preschool education. As an important training method for preschool teachers, higher vocational colleges provide a large number of talents for preschool education. Among them, the five-year consistent production is an important training mode for the preschool education major in higher vocational education, and its curriculum setting directly affects the teaching and the cultivation of talents, as shown in the following formula:

(4) $$\begin{array}{c} d_{i}={\left(X-X_{i}\right)}^{2}+{\left(Y-Y_{i}\right)}^{2}. \end{array}$$

In order to gain a detailed understanding of the actual situation of the hand-made curriculum in the five-year consistent system of preschool education and also to ensure that the research has practical application value, this paper, as a case study institution, takes the situation of the five-year consistent system of preschool education hand-made curriculum in the H College as a case study. For the research object of this article, according to its curriculum standards, curriculum teaching plan, and other relevant materials, the curriculum objectives, curriculum structure, curriculum content text content are listed, and the current situation of the text setting is understood. Five-year consistent preschool education students will issue papers, analyze the data, and understand the students' recognition of the hand-made curriculum; through interviews with teachers, they understand the actual situation of the hand-made curriculum and implementation, as follows:

(5) $$\begin{array}{c} \text{foundation}=\sum_{i=1}^{n}\left|X_{i}-Y_{i}\right|. \end{array}$$

## 3. Handmade Process for Preschool Professionals

Curriculum objectives and teaching objectives have a mutually unified relationship. From the perspective of teachers and students or from the process of curriculum implementation, curriculum objectives are also teaching objectives, and the two are consistent and unified. Criteria for the division of teaching objectives can be used in the division of overall curriculum objectives. According to the classification method of teaching objectives of Bloom et al., the teaching objectives are divided into target classification in the cognitive domain, target classification in the sensory domain, and target classification in the motor skills domain. Accordingly, curriculum objectives are usually divided into three categories: knowledge objectives, skill objectives, and emotional objectives.

According to the text content of the general objective of the hand-made curriculum, the curriculum objectives are divided into knowledge objectives and ability objectives, of which the ability objective is the skill objective. Through observation, it is found that the division of skills curriculum objectives is inaccurate, mainly in the following two aspects. First, the expression of knowledge objectives contains the content of skills objectives. For example, be able to skillfully use basic hand tools and simple materials for handcraft, and have a certain level of material selection, color matching, compositional balance, and use of technique. Secondly, the expression of skill goals also contains the content of emotional goals. This course is of great help in cultivating students' conscientiousness, patience, and meticulous quality, improving their aesthetic ability, hands-on ability, and artistic creation ability, and laying a solid foundation for their future manual teaching. Among them, the description of cultivating students' seriousness, patience, and meticulous quality should belong to the content of emotional goals, as the following formula:

(6) $$\begin{array}{c} \text{occupation}=\underset{k⟶\infty }{\lim}{\left(X_{i}-Y_{i}\right)}^{1/k}. \end{array}$$

As a core skill course, handcrafted courses are expressed in the form of achievement goals, a short statement that accurately describes what an individual can do in a course to demonstrate the individual's mastery of the task after the learning activity. The analysis found that in the expression of situational goals, the five parts of the content appeared many times to understand, master, and understand such verbs to describe the state, such as paper-cutting situational learning curriculum goals and understanding the history and development of paper-cutting. What is understanding? What is the judging standard for understanding? To understand the artistic characteristics and basic types of paper-cutting, it is necessary to understand the paper-cutting process based on the use of a certain basic type. The use of descriptive verbs such as mastery is not standard, which makes the overall expression of the course objectives unclear. The inability to clearly measure the degree of understanding and mastery greatly weakens the normative and scientific nature of curriculum goal setting. At the same time, in the course of curriculum implementation, due to the differences in teachers' own abilities, the understanding of curriculum goals such as understanding and mastery is not clear. There are certain problems in the realization of the course objectives, as follows:

(7) $$\begin{array}{c} \text{utilization}=\text{max}\left(X-X_{i},Y-Y_{i}\right). \end{array}$$

As the basic course of manual courses, the hand-making course can not only cultivates students' manual ability but also cultivates students' innovative ability. At the same time, the hand-made course is an art skill course, which can also improve students' art literacy and aesthetic ability through learning. This requires that both the basic craftsmanship skills that students should master and the content of the students' craftsmanship innovation ability should be reflected in the handcraft curriculum. However, through the investigation, it was found that the curriculum objectives of the hand-made course learning situation focused on the practice of craftsmanship and lacked the goal of inspiring and innovative ability training for students. For example, take the origami course goal as an example; the main emphasis in the course goal is to master the basic skills of origami, understand and master the folding method of flowers and small animals, and combine them. In the statement of the course objectives, there is no relevant explanation about the requirement of origami to cultivate students' innovative ability, as the following formula:

(8) $$\begin{array}{c} \text{skill}\_\text{scores}=\frac{\langle X_{i},Y_{i}\rangle }{\left\|X_{i}\right\|\left\|Y_{i}\right\|}. \end{array}$$

Through the investigation, it is found that the content of the current hand-made courses is mainly arranged according to the content of the teaching materials and teachers' experience, and the setting of the course content cannot be updated in time according to the needs of the job position, and the update of new craftsmanship techniques is slow. It reflects the separation between the specific curriculum content setting and the actual job requirements. For example, compiling the curriculum content is difficult to use in actual kindergarten teaching activities. However, in the five-year system, curriculum content still exists in the handcrafted curriculum content setting. The content of the hand-made course cannot be updated in time, and it is difficult to adjust the content of the course according to the students' future work needs over time, as the following formula:

(9) $$\begin{array}{c} \text{investigation}=\sqrt{\left(X-X_{i}\right)}+\sqrt{\left(Y-Y_{i}\right)}. \end{array}$$

The setting of manual course content not only needs to consider the needs of teaching content but also needs to consider the needs of students. The needs of students mainly include two aspects: first, to meet the needs of students for self-learning. Students' self-learning needs refer to the needs of students to learn and expand the same type of handicraft techniques after class after mastering a hand-made technique. Second, to meet the needs of students in the future work, the technical skills in the hand-made course content can meet the needs of the job. The research shows that students think that the five parts of paper-cutting, origami, pasting painting, masonry, and knitting can neither meet the needs of future work nor the current self-study needs, as the following formula:

(10) $$\begin{array}{c} \text{manual\_score}=\text{min}\left(\left|X-X_{i}\right|,\left|Y-Y_{i}\right|\right). \end{array}$$

## 4. Optimization Analysis of Intangible Cultural Heritage Digital Resource Service System

### 4.1. The Digital Coverage of Intangible Cultural Heritage Is Low, and There Is a Lack of a Complete Digital Resource Service Platform

Compared with such a rich number of intangible cultural heritage, the existing digital resources are not complete compared to the intangible cultural heritage projects themselves and can only meet the needs of project declaration. In addition, judging from the construction of existing resources, there is still a long way to go to improve the service platform for digital resources of intangible cultural heritage. The calculation of digital resources is shown in formula 11.

(11) $$\begin{array}{c} \left\{\begin{array}{c} cx_{l}=f\frac{X_{p}}{Z_{p}},\\ cx_{r}=fkl\frac{X_{p}-T}{Z_{p}},\\ \text{overall}\_y=fkk\frac{Y_{p}}{Z_{p}}. \end{array}\right) \end{array}$$

At present, digital resources have problems such as single type, simple content, and low utilization rate of new technologies. The quality of intangible cultural heritage digital resources at the municipal level is even more uneven, and the regional differences are large. In addition, many collected data resources cannot be publicly provided to the public, making it difficult to meet the public's viewing needs. The project lacks a standard specification system based on top-level design and lacks systematic, scientific, and reasonable ideas and solutions for digital protection.

### 4.2. Lack of Standard Specification System Based on Top-Level Design

The research object has not formed a unified standard and normative system for digital protection work for the time being. There is a lack of unified, institutionalized, and standardized digital collection standards for intangible cultural heritage, and the digital resources collected are fragmented, with insufficient professionalism and low content coverage and lack of systematic standards for metadata, classification, and format of digital, as follows:

(12) $$\begin{array}{c} \left[\begin{array}{c} H\\ W\\ V \end{array}\right]=\left[\begin{array}{ccc} \frac{1}{dxy} & 0 & u_{0}\\ 0 & \frac{1}{dzy} & v_{0}\\ 0 & 0 & \frac{1}{d\text{x}z} \end{array}\right]\left[\begin{array}{c} x\\ y\\ 1 \end{array}\right]. \end{array}$$

The quality of resources is uneven; lack of business standards for digital resource storage, access, sharing, etc. cannot realize the processing, storage, and integration of digital resources, resulting in waste of resources and inconvenience to resource services. In the final analysis, the lack of a standard and normative system based on top-level design has resulted in large differences in the intangible cultural heritage databases that have been built and difficulty in data integration, which reduces the service value and efficiency of digital resources, resulting in slow progress in the service of intangible cultural heritage digital resources in our research objective.

### 4.3. Insufficient Funds and Publicity Measures and Lack of Enthusiasm for Public Participation

There is still some gap between the investment in the special protection of intangible cultural heritage and the demand. The annual investment is expected to be 40 million, but the actual annual investment in intangible cultural heritage is only 20 million. Therefore, we can only choose to invest in key protected intangible cultural heritage projects, and other projects can only suspend work. There are not enough and stable funds to develop resource services, which aggravates the possibility of service work being stagnant. In addition, the daily publicity is not enough, and the public participation is low. Due to the lack of government incentives, conventional publicity methods are still adopted, and the connotation of intangible cultural heritage is insufficiently explored, as the following formula.

(13) $$\begin{array}{c} H=-\int_{0}^{1}\int_{0}^{1}P_{\text{i}1\text{,i}2}\left({\text{i}}_{1}{\text{,i}}_{2}\right)\log\;P_{i1,i2}\left(i_{1},i_{2}\right). \end{array}$$

As a result, the public still regards intangible cultural heritage resources as tourism and entertainment projects, lacks active participation and enthusiasm, and is not closely connected with the public. To sum up, at present, the construction and service of Jiangsu intangible cultural heritage digital resources are still in the process of exploration, and a complete service system has not yet been formed. The fundamental reason is that the digital protection mechanism of intangible cultural heritage at the national level is imperfect and the standardization work is backward, which leads to the wrong reference of lower-level governments, and it is difficult for the lower-level government to be effective. Second, there is still a lack of user-oriented and demand-oriented research, relying only on the policy planning of the higher-level government to formulate service goals. Third, there is a lack of a digital protection system covering the whole province. In the face of the current situation of multiple management, the established intangible cultural heritage digital resource services are quite different, and there are difficulties in docking and integration, which will naturally lead to the slow progress of the intangible cultural heritage digital resource services in our research.

### 4.4. Experiment Results

Regarding the composition of the intangible cultural heritage digital resource service, the survey result is shown in Figure 1, which shows that in addition to 20% of the respondents who said they were unwilling to use it, 65% of the respondents said they were willing to use it, and the proportion of respondents in some places who agreed is higher, and 40% of the respondents said that it depends on the content of the resource and the level of service. It shows that the demand for providing intangible cultural heritage digital resource services does exist, and it should meet their needs and provide high-level resource services. Moreover, in order to increase the use of service objects and their preference for service channels of intangible cultural heritage digital resources, 45.02% and 50.86% of the respondents expressed their willingness to use the service channels of public cultural institutions' self-built databases and government intangible cultural heritage websites. It shows that compared with open network resources, users are more willing to use digital resource services provided by government departments and related cultural institutions.

Figure 2 shows the specific classification results of material cultural heritage. Content enrichment requires rich and diverse contents and service methods of intangible cultural heritage digital resources. The first thing to do is to speed up the digitization of intangible cultural heritage resources. Government departments organize participating institutions to carry out the collection of intangible cultural heritage digital resources and the digitization of physical resources. Secondly, build an intangible cultural heritage database group covering a variety of media types, gradually carry out the construction of intangible cultural heritage digital resources, and strive to build a city's intangible cultural heritage special website in the short term. Finally, the established resource services should focus on enriching the way of digital resource services, realize digital resource services at different levels such as basic services, knowledge-based services, and personalized customized services, and pay attention to the in-depth development of knowledge. Count invention is shown in Figure 3.

The results of the survey in Figure 3 show that the reasons for the respondents to use intangible cultural heritage digital resource services are diverse: 7196 respondents are for acquiring knowledge and skills, and 97% and 98% are for personal hobbies. For leisure and entertainment, many respondents use intangible cultural heritage digital resource services because of academic research, work, or assignments. The main reason for respondents in Nanjing and Suzhou to use the service was to acquire knowledge and skills, while in Xuzhou, it was mostly for academic research. As for the reasons for not using intangible cultural heritage digital resource services, 98.5% of the respondents indicated that there is no such demand for the time being, and 98.4% of users did not know that digital resource services are provided. This shows that if we want to develop intangible cultural heritage digital resource services, we must strengthen the promotion work for service objects with explicit and implicit needs, so that they can fully understand the intangible cultural heritage digital resource services and increase their enthusiasm for use.

How does the public obtain digital resource services for intangible cultural heritage? The survey results are shown in Figure 4, which show that respondents generally use intangible cultural heritage websites and digital libraries to obtain resources, accounting for 74% and 80%, respectively. There are significantly more respondents to the special website on cultural heritage, which is related to the relatively complete construction of the intangible cultural heritage website and complete service functions. It shows that it is very necessary to establish an intangible cultural heritage website in this area, which can facilitate users to obtain the desired digital resources and services more comprehensively and quickly.

## 5. Conclusion

The research of this paper provides research ideas for the protection of intangible cultural heritage. Although this paper has obtained some meaningful research conclusions, there are still some shortcomings, which have a certain impact on the research conclusions. First of all, due to the lack of practical environment, this paper can only conduct theoretical discussions on the basis of previous research and practice, and it is still in the preliminary stage of peeking at the leopard. The construction of the intangible cultural heritage digital resource service system is a relatively realistic problem, and the effectiveness and operability of its service elements, model framework, construction ideas, and implementation paths need time to be verified. Secondly, there are certain deficiencies in the questionnaire survey in this paper. Compared with the huge sample size, the sample size of the questionnaire is insufficient; the content design of the questionnaire is relatively simple, and the investigation is not deep enough, so it is difficult to comprehensively and deeply reflect the actual needs of digital resource services for intangible cultural heritage. The third is that the proposed optimization strategy for the digital resource service system for intangible cultural heritage lacks interviews and confirmations from government departments, and the opinions seem to be “castles in the air.” This paper hopes to draw some valuable insights from it, provide suggestions for future theoretical research and practical work in this field, and help the construction of our country's intangible cultural heritage digital resource service system to achieve more brilliant results.

## Figures and Tables

**Figure 1:** The ratio of different types of resources.

**Figure 2:** Cultural heritage classification from UNESCO-21.

**Figure 3:** Count invention.

**Figure 4:** Channel sources for using intangible cultural heritage materials.

## Data Availability

The data used to support the findings of this study are available from the corresponding author upon request.
